This article has been retracted.

# Efficacy of Duhuo Jisheng Decoction in Treating Ankylosing Spondylitis: Clinical Evidence and Potential Mechanisms

**DOI:** 10.1155/2022/3305773

**Published:** 2022-04-04

**Authors:** Yi Wang, Zhihua Zhou, Li Chen, Xiangwei He, Hui Li, Yingru Huang, Yu Pu

**Affiliations:** ^1^Department of Orthopedic, Chongqing Jiangbei hospital of Traditional Chinese Medicine, Chongqing 400020, China; ^2^Chongqing Key Laboratory of Traditional Chinese Medicine for Prevention and Cure of Metabolic Diseases, Chongqing Medical University, College of Traditional Chinese Medicine, Chongqing 400016, China

## Abstract

**Background:**

Duhuo Jisheng Decoction (DHJSD) is an ancient compound widely used in the treatment of ankylosing spondylitis (AS). However, its efficacy is controversial, and its mechanism of action is not clear enough. Using meta-analysis and network pharmacology, our study evaluated the clinical efficacy of DHJSD in the treatment of AS and explored its mechanisms of action.

**Methods:**

We searched medical databases, including Embase, PubMed, the China National Knowledge Infrastructure databases, Wanfang, and the Chinese Scientific Journal Database, to identify studies that met the inclusion criteria. RevMan 5.3 software was used for the meta-analysis. The compounds and the potential protein targets of DHJSD were obtained from the Traditional Chinese Medicine Systems Pharmacology (TCMSP) database and analysis platform. AS was treated as a search query in the NCBI, PharmGKB, TTD, DrugBank, and OMIM databases to obtain disease-related genes. The overlapping targets of DHJSD and AS were identified, and then Gene Ontology functional enrichment and Kyoto Encyclopedia of Genes and Genomes enrichment analyses were performed. Cytoscape was employed to construct a drug-compound-target network and a protein-protein interaction (PPI) network. CytoHubba was utilized to select the hub genes.

**Results:**

A total of 10 studies involving 860 participants were included in the meta-analysis. Compared with the control, DHJSD treatment significantly improved clinical symptoms; reduced the erythrocyte sedimentation rate (ESR), the C-reactive protein (CPR), and interleukin 6 (IL-6) levels; increased the degree of motion of the chest; reduced the visual analog scale (VAS) pain score; reduced Schober's test values; reduced the finger-to-floor distance; reduced the duration of morning stiffness. However, the differences were not statistically significant in the Bath Ankylosing Spondylitis Functional Index scores, the Bath Ankylosing Spondylitis Disease Activity Index scores, the bone Gla-containing protein (BGP) levels, or the bone alkaline phosphatase (BALP) levels. In terms of adverse events, DHJSD treatment of AS reduced the incidence of gastrointestinal events, the incidence of skin events, and the incidence of abnormal liver function; however, there was no statistically significant reduction in the incidence of adverse renal function events. Subgroup analysis showed that in the treatment of AS, the clinical effect of DHJSD for AS was better than that of the controls for both treatment durations, ≤2 months and >2 months. A total of 178 active compounds and 47 related potential targets were identified for DHJSD in the treatment of AS, including four hub genes (CXCL8, PTGS2, VEGFA, and STAT3). The core active ingredients of DHJSD in the treatment of AS were mainly quercetin, kaempferol, licochalcone A, and isorhamnetin. DHJSD treatment of AS-related pathways mainly involved the IL-17 signaling pathway, the TNF signaling pathway, and the rheumatoid arthritis signaling pathway.

**Conclusion:**

The above results suggest that DHJSD acts on AS through multiple targets, components, and pathways with significant clinical efficacy. Future studies may further explore the active components of DHJSD.

## 1. Introduction

Ankylosing spondylitis is a chronic inflammatory disease that mainly affects large joints, such as the sacroiliac joint and the spine, but it can damage the surrounding small joints as well. It can cause spinal stiffness and deformity. The disability rate is as high as 30%, which seriously affects the quality of life of patients [1, 2].

At present, this disease still cannot be cured. Treatment is used mainly to control the clinical symptoms, slow down disease progression, and improve the patient's prognosis. Western medicines are mainly antirheumatic drugs, such as NSAIDs and glucocorticoids [3–5]. However, long-term use of Western drugs has its disadvantages, such as adverse gastrointestinal reactions, liver and kidney damage, the worsening of the condition after drug withdrawal, and high costs [6, 7].

Ankylosing spondylitis falls into the categories of “nephroparalysis” and “bone impediment” in traditional Chinese medicine (TCM) [8–10]. In the treatment of ankylosing spondylitis, Chinese medicine mainly focuses on replenishing the liver and kidneys, replenishing qi and blood, dispelling rheumatism, and relieving arthralgia [11, 12]. The clinical application of TCM in the treatment of ankylosing spondylitis is based on a wealth of experience. It has the advantages of providing definite curative effects with few adverse reactions, and its application prospects are good.

Duhuo Jisheng Decoction (DHJSD) is a classic prescription commonly used to treat liver and kidney deficiency, deficiency of essence and blood, and chronic arthralgia. It has the functions of nourishing the liver and kidneys, nourishing essence and blood, strengthening muscles and bones, removing dampness, and relieving arthralgia [13, 14].

DHJSD is mainly composed of Du Huo (Radix Angelicae Pubescentis), Sang Ji Sheng (Herba Taxilli), Qin Jiao (Radix Gentianae Macrophyllae), Fang Feng (Radix Saposhnikoviae), Xi Xin (Herba Asari), Fu Ling (Poria Cocos), Chuan Xiong (Rhizoma Chuanxiong), Bai Shao (Radix Paeoniae Alba), Du Zhong (Cortex *Eucommiae Ulmoidis*), Ren Shen (Panax Ginseng), Gan Cao (Radix Glycyrrhizae), Dang Gui (Radix Angelicae Sinensis), Niu Xi (Radix Achyranthis Bidentatae), Shu Di Huang (Radix Rehmanniae Preparata), and Rou Gui (Cortex Cinnamomi) [13]. There are currently many clinical randomized controlled trials reporting AS treated by DHJSD, but the sample sizes are small, and the research results offer limited clinical guidance. Therefore, this study evaluated the efficacy and safety of DHJSD in the treatment of AS by meta-analysis and provided evidence-based guidance for DHJSD's clinical application. At present, network pharmacology analysis has been widely used to evaluate the interaction between proteins and molecules in biological systems and to study the mechanism of action of Chinese medicine. This combination of classical pharmacology and systematic pharmacology analysis may provide a better strategy for determining new therapeutic uses of, and the mechanisms in, traditional Chinese medicine. Therefore, we used the network pharmacology research method to predict the effective components, targets, and key pathways of DHJSD in the treatment of AS and thus to explain its mechanism of action.

## 2. Methods

### 2.1. Search Strategy

A systematic search of PubMed, Embase, the China National Knowledge Infrastructure databases, Wanfang, and the Chinese Scientific Journal Database was conducted from inception to June 30, 2021, with no language restriction. Randomized controlled trials (RCTs) that involved the use of DHJSD for the treatment of AS were collected. The keywords used were as follows: Duhuo Jisheng Decoction, Duhuo Jisheng Tang, DHJSD, Ankylosing Spondylitis, and Bechterew Disease. Furthermore, we manually searched the reference lists of the included studies for additional studies.

### 2.2. Inclusion and Exclusion Criteria

The inclusion criteria included the following:

- Patients with a clear diagnosis of AS; no restrictions on race, sex, or age were imposed
- RCTs
- Control group for Western medicine treatment and experimental group for treatment with DHJSD based on the control group
- One or more of the following outcome indicators had to be present: (1) primary outcome: clinical efficacy; (2) secondary outcomes: Bath Ankylosing Spondylitis Functional Index (BASFI), Bath Ankylosing Spondylitis Disease Activity Index (BASDAI), Visual Analog Scale (VAS) pain score, Finger-to-floor distance, morning stiffness duration, degree of motion of chest, Schober's test values, Erythrocyte Sedimentation Rate (ESR), C-reactive protein (CPR), bone alkaline phosphatase (BALP), interleukin 6 (IL-6), bone Gla-containing protein (BGP), and adverse events

The exclusion criteria included the following:

- Republished studies
- Non-RCTs
- Experiments on animals
- Studies lacking literature data
- Reviews, conference reports, system reviews, protocols, or abstracts

### 2.3. Data Collection and Quality Assessment

All the retrieved search results were summarized and imported into Endnote, which was used to delete duplicate searches. By reading the title of the article and the abstract, the literature that did not meet the inclusion criteria was preliminarily excluded. The full text of the literature that met the inclusion criteria after the initial screening was downloaded, and two independent authors read the full text of each source carefully and cross-checked its content against the inclusion/exclusion criteria. For controversial literature, the two authors discussed their differences and either reached a resolution or asked the third author to evaluate the article and make a decision. The data extracted from the articles included the following: (1) general information: the name of the first author, research time, sample size, gender, and age; (2) research design method: random allocation of specific methods; blinding; loss to follow-up; withdrawal cases in the research analysis; (3) treatment status: the specific drug name, dose, frequency, course of treatment, and route of administration used in the treatment group and the control group; (4) outcome indicators: clinical effective rate and BASFI, BASDAI, and VAS scores. If some studies lacked data that affected the final statistical analysis, the author was contacted, as necessary, to supplement it.

RCTs were evaluated by the researchers based on the Cochrane risk bias assessment tool. Assessments included random assignment methods, allocation concealment, blinding methods, missing outcome data, selecting result reports, and other biases.

### 2.4. Data Synthesis and Statistical Analysis

Meta-analysis was performed with RevMan 5.3 software. Dichotomous data were reported as risk ratios (RRs) with 95% confidence intervals. Continuous data were calculated as the standard mean difference (SMD) with associated 95% CIs. When the heterogeneity was too large or if we were unable to find the data source, the meta-analysis was abandoned, and only descriptive analysis was performed. A subgroup analysis was performed according to the course of treatment (≤2 months and >2 months). The sensitivity of each index was analyzed with the elimination method to test the stability of the results. If no fewer than ten articles were included, then Begg's funnel plot and Egger's regression analysis were used to test for publication bias.

### 2.5. Network Pharmacology-Based Prediction of the Potential Actions of DHJSD on AS

#### 2.5.1. Screening of Active Compounds in DHJSD

Du Huo, Qin Jiao, Sang Ji Sheng, Fang Feng, Fu Ling, Xi Xin, Chuan Xiong, Bai Shao, Du Zhong, Ren Shen, Gan Cao, Dang Gui, Niu Xi, Shu Di Huang, and Rou Gui are monarchs and minister herbs, which are regarded as the main active herbs in DHJSD that have the Latin names of Radix Angelicae Pubescentis, Herba Taxilli, Radix Gentianae Macrophyllae, Radix *Saposhnikoviae*, Herba Asari, Poria Cocos, Rhizoma Chuanxiong, Radix Paeoniae Alba, Cortex *Eucommiae ulmoidis*, Panax Ginseng, Radix Glycyrrhizae, Radix Angelicae Sinensis, Radix Achyranthis Biatae, Radix *Rehmanniae* Preax Ginsta, and Radix Glycyrrhizae, respectively.

The active chemical components of DHJSD's component drugs were searched using the TCMSP, Version: 2.3, https://tcmspw.com/tcmsp.php database.

#### 2.5.2. Screening of the Target Genes of Active Compounds

The active ingredients screened in DHJSD were searched through the TCMSP platform to find their corresponding target proteins. The UniProt database was used to query the gene names corresponding to the target proteins, merge duplicate targets of action, and delete proteins without corresponding gene names.

#### 2.5.3. Acquisition of AS-Related Target Genes and Identification of Candidate Target Genes of DHJSD Acting on AS

“Ankylosing Spondylitis” was used as the keyword search term in the National Center for Biotechnology Information (NCBI), Online Mendelian Inheritance in Man (OMIM), Pharmacogenomics Knowledgebase (PharmGKB), Therapeutic Target Database (TTD), and DrugBank.

#### 2.5.4. Construction of the Medicine-Compound-Target Network

Cytoscape 3.8.0 software was used to build a “drug-compound-target” network and to analyze compounds and targets. Disease-drug names, active ingredients, and targets are represented by “nodes,” and the interrelationships between nodes are represented by “edges.”

#### 2.5.5. Construction of the Protein-Protein Interaction (PPI) Network and Selection of Key Targets

We imported the potential targets of DHJSD in treating AS into the STRING database, selected the species as “Homo sapiens,” selected the minimum required interaction score as medium confidence (0.400), removed the free nodes, obtained the protein interaction information, and saved it in “TSV” format. The “TSV” file was imported into Cytoscape 3.8.0 to draw a protein-protein interaction (PPI) network. We analyzed the nodes in the network through the plug-in CytoNCA. We calculated the betweenness centrality (BC), closeness centrality (CC), degree centrality (DC), eigenvector centrality (EC), local average connectivity-based method centrality (LAC), and network centrality (NC) of each node in the network. Nodes with DC ≥ median, CC ≥ median, BC ≥ median, EC ≥ median, LAC ≥ median, and NC ≥ median were selected, and the first screening was completed. We established a subnetwork and once again used the plug-in CytoNCA to calculate the DC, BC, CC, EC, LAC, and NC of the nodes in the subnetwork and to filter out DC ≥ median, CC ≥ median, BC ≥ median, and EC ≥ median for nodes with LAC ≥ median and NC ≥ median; thus, we complete the second screening. We drew a flowchart to visualize the screening process.

#### 2.5.6. GO Function Enrichment and KEGG Pathway Enrichment Analysis

R 4.1.0 software and its “org.Hs.eg.db” package were used to obtain the ID of the intersection target. Then, program packages such as “clusterProfiler” were used to perform GO function enrichment analysis on the target and screen out the top 10 functional categories of biological process (BP), cellular component (CC), and molecular function (MF) and to draw them into a histogram. Then, KEGG enrichment analysis was performed on the target, the first 20 KEGG pathways were selected, and a histogram was drawn. *P* < 0.05 was the screening condition.

## 3. Results

### 3.1. Meta-Analysis

#### 3.1.1. Literature Search Results

A total of 396 studies were searched, and 249 studies were obtained after removing duplicates. After screening, ten papers were finally included. The literature screening process is shown in Figure S1. A total of 860 patients with AS were included in the ten publications [15–24], including 434 cases in the experimental group and 424 cases in the control group. The basic characteristics of the included literature are shown in Table 1. The results of the risk of bias evaluation are shown in Figure 1.

#### 3.1.2. Clinical Efficacy

The clinical effective rate was compared among the ten studies, with 434 cases in the experimental group and 424 cases in the control group. There was some heterogeneity (heterozygosity test: *P*=0.02, I2 = 53%). When the random effect model was used to merge RR values, the pooled RR was 1.30 (95% CI: 1.16–1.44, *P* < 0.00001). This indicated that the clinical effective rate was significantly higher in the experimental group than that in the control group (Figure S2 and Table 2).

#### 3.1.3. BASFI

Four studies reported BASFI scores for 189 cases in the experimental group and 196 cases in the control group. There was heterogeneity across the studies (heterozygosity test: *P* < 0.00001, I2 = 97%). The random-effects model combined SMD, and the pooled SMD was −0.46 (95% CI: 1.77–0.85, *P*=0.49). This indicated that the difference in BASFI scores between the experimental and control groups after treatment was not statistically significant (Figure S3 and Table 2).

#### 3.1.4. BASDAI

Three studies reported BASDAI scores for 139 cases in the experimental group and 146 cases in the control group. There was heterogeneity across the studies (heterozygosity test: *P* < 0.00001, I2 = 97%). The random-effects model combined SMD, and the pooled SMD was −0.36 (95% CI: −1.95–1.23, *P*=0.66). These results indicated that the difference in BASDAI scores between the experimental and control groups after treatment was not statistically significant (Figure S4 and Table 2).

#### 3.1.5. VAS Pain Score

Six studies reported VAS pain scores for a total of 515 patients with AS. There was heterogeneity across the studies (heterozygosity test: *P*=0.0003, I2 = 97%). The random-effects model combined SMD, and the pooled SMD was -0.79 (95% CI: −1.19 to −0.40, *P* < 0.0001). Compared with the control groups, the DHJSD treatment groups were associated with reduced VAS pain scores (Figure S5 and Table 2).

#### 3.1.6. Finger-to-Floor Distance

Five studies reported the outcomes of finger-to-floor distance for 481 patients with AS. There was heterogeneity across the studies (heterozygosity test: *P* < 0.00001, I2 = 97%). The random-effects model combined SMD, and the pooled SMD was −1.55 (95% CI: −2.66 to −0.44, *P*=0.006). Compared with the control groups, the DHJSD treatment groups were associated with reduced finger-to-floor distance (Figures S6 and Table 2).

#### 3.1.7. Morning Stiffness Duration

Three studies reported the outcomes of morning stiffness duration for 230 patients with AS. There was heterogeneity across studies (heterozygosity test: *P* < 0.0001, I2 = 91%). The random-effects model combined SMD, and the pooled SMD was−1.23 (95% CI: −2.21 to −0.25, *P*=0.01). Compared with the control groups, the DHJSD treatment groups were associated with reduced morning stiffness time (Figure S7 and Table 2).

#### 3.1.8. Degree of Motion of Chest

Three studies reported *r*, the outcomes of the degree of motion of the chest for 285 patients with AS. The three studies had homogeneity (heterozygosity test: *P*=0.80, I2 = 0%). The fixed-effects model combined SMD, and the pooled SMD was 0.24 (95% CI: 0.01–0.47, *P*=0.04). Compared with the control groups, the DHJSD treatment groups were associated with an increased degree of motion of the chest (Figure S8 and Table 2).

#### 3.1.9. Schober's Test Values

Three studies reported Schober's test values for 321 patients with AS. The three studies had homogeneity (heterozygosity test: *P*=0.24, I2 = 31%). The fixed-effects model combined SMD, and the pooled SMD was 0.23 (95% CI: 0.01–0.45, *P*=0.04). Compared with the control groups, the DHJSD treatment groups were associated with increased Schober's test values (Figure S9 and Table 2).

#### 3.1.10. ESR

Nine studies reported the outcomes of ESR levels for 800 patients with AS. There was heterogeneity across the studies (heterozygosity test: *P* < 0.00001, I2 = 94%). The random-effects model combined SMD, and the pooled SMD was −1.07 (95% CI: −1.69 to −0.46, *P*=0.0006). Compared with the control groups, the DHJSD treatment groups were associated with reduced ESR levels (Figure S10 and Table 2).

#### 3.1.11. CPR

Seven studies reported the outcomes of CPR levels for 582 patients with AS. There was heterogeneity across the studies (heterozygosity test: *P* < 0.00001, I2 = 97%). The random-effects model combined SMD, and the pooled SMD was −2.31 (95% CI: −3.52 to −1.10, *P*=0.0002). Compared with the control groups, the DHJSD treatment groups were associated with reduced CPR levels (Figure S11 and Table 2).

#### 3.1.12. BALP

Two studies reported the outcomes of BALP levels for 211 patients with AS. There was heterogeneity across the studies (heterozygosity test: *P*=0.05, I2 = 74%). The random-effects model combined SMD, and the pooled SMD was 0.18 (95% CI: −0.36 to −0.71, *P*=0.51). This indicated that the difference in BALP levels between the experimental groups and the control groups after treatment was not statistically significant (Figure S12 and Table 2).

#### 3.1.13. IL-6

Two studies reported the outcomes of IL-6 levels for 211 patients with AS. There was heterogeneity across the studies (heterozygosity test: *P* < 0.0001, I2 = 94%). The random-effects model combined SMD, and the pooled SMD was −1.72 (95% CI: −3.06 to −0.38, *P*=0.01). Compared with the control groups, the DHJSD treatment groups were associated with reduced IL-6 levels (Figure S13 and Table 2).

#### 3.1.14. BGP

Two studies reported the outcomes of BGP levels for 211 patients with AS. There was heterogeneity across the studies (heterozygosity test: *P* < 0.00001, I2 = 99%). The random-effects model combined SMD, and the pooled SMD was 3.14 (95% CI: −1.62–7.89, *P*=0.20). This indicated that the difference in BGP levels between the experimental groups and the control groups after treatment was not statistically significant (Figure S14 and Table 2).

#### 3.1.15. Adverse Events

Five studies reported the incidence of gastrointestinal events associated with DHJSD in AS. The five studies had homogeneity (heterozygosity test: *P*=0.62, I2 = 0%). When the fixed effect model was used to merge RR values, the pooled RR was 0.27 (95% CI: 0.13–0.54, *P*=0.0002). This indicated that the incidence of gastrointestinal events was significantly lower in the experimental groups than it was in the control groups (Figure S15, Table 2).

Five studies reported the incidence of skin events associated with DHJSD in AS. The five studies had homogeneity (heterozygosity test: *P*=0.88, I2 = 0%). When the fixed-effects model was used to merge RR values, the pooled RR was 0.13 (95% CI: 0.03–0.48, *P*=0.002). This indicated that the incidence of skin events was significantly lower in the experimental groups than it was in the control groups (Figure S16 and Table 2).

Six studies reported the incidence of the abnormal liver function of DHJSD in AS. The six studies had homogeneity (heterozygosity test: *P*=0.85, I2 = 0%). When the fixed-effects model was used to merge RR values, the pooled RR was 0.28 (95% CI: 0.11–0.67, *P*=0.004). This indicated that the incidence of abnormal liver function was significantly lower in the experimental groups than it was in the control groups (Figure S17 and Table 2).

Three studies reported the incidence of abnormal renal function associated with DHJSD in AS. The three studies had homogeneity (heterozygosity test: *P*=0.96, I2 = 0%). When the fixed effect model was used to merge RR values, the pooled RR was 0.29 (95% CI: 0.05–1.72, *P*=0.17). This indicated that the incidence of abnormal renal function was not significantly different between the experimental groups and the control groups (Figure S18 and Table 2).

#### 3.1.16. Subgroup Analysis

According to the course of treatment, studies were divided into two subgroups (≤2 months and >2 months) to analyze the clinical effective rates in AS patients. The results of subgroup analysis showed that the clinical effective rates of the experimental groups were higher than those of the control groups, regardless of whether the treatment course was ≤2 months (RR = 1.20, 95% CI (1.09–1.31), *P*=0.0001) or >2 months (RR = 1.40, 95% CI (1.16–1.70), *P*=0.0006), and the difference was statistically significant (Figure S19).

#### 3.1.17. Sensitivity Analysis

Sensitivity analysis of the clinical effective rate showed that the results of this meta-analysis were stable (Figure S20).

#### 3.1.18. Publication Bias

Begg's funnel plot and Egger's test were performed to evaluate publication bias (Figure S21). The results showed a statistically significant difference in the clinical effective rate (Begg's test: *P*=0.012; Egger's test: *P*=0.023).

### 3.2. Network Pharmacology

#### 3.2.1. “DHJSD” Medicinal Chemical Constituents and Related Targets

By querying the TCMSP database, after screening with OB ≥ 30% and DL ≥ 0.18, a total of 179 active compounds were obtained, of which seven compounds were from Radix Paeoniae Alba, six were from Rhizoma Chuanxiong, three compounds were from Radix Angelicae Sinensis, eight were from Radix Angelicae Pubescentis, 25 were from Cortex *Eucommiae Ulmoides*, 18 were from Radix Saposhnikoviae, six were from Poria Cocos, 88 were from Radix Glycyrrhizae, 16 were from Radix Achyranthis Bidentatae, two were from Radix Gentianae Macrophyllae, 17 were from Panax Ginseng, two were from Herba Taxilli, ten were from Cortex Cinnamomi, three were from Radix Rehmanniae Preparata, and seven were from Radix Herba Asari. In addition, based on these compounds, 262 predicted targets of DHJSD were found. A total of 178 active ingredients were extracted from the TCMSP database. Information on active compounds in DHJSD and the number of corresponding targets are shown in Table S1.

#### 3.2.2. “Ankylosing Spondylitis” Disease Target Search Results

By searching the NCBI, OMIM, PharmGKB, TTD, and DrugBank databases, a total of 398 AS-related targets were obtained.

#### 3.2.3. Drug-Disease Intersection Target, Venn Diagram, and Drug-Compound-Target Gene Network

The targets of DHJSD and AS-related targets were crossed, and 47 crossed targets were obtained; that is, there were 47 potential targets for DHJSD in the treatment of AS. The results are shown in Figure S22. Cytoscape 3.8.0 software was used to draw the “drug-compound-target gene” regulatory network. The DHJSD medicinal components were matched with the 47 target points obtained from the screening. As shown in Figure S23, the network contains 633 nodes and 30005 edges. From the overall characteristics of the network, we found that among the 153 DHJSD compounds, one compound corresponded to multiple targets, and one target corresponded to multiple compounds. The larger the node is, the larger the network value of the target is. It can be seen from the regulatory network that the most connected chemical substance is quercetin, which interacts with 34 targets, followed by kaempferol, which interacts with 15 targets; licochalcone interacts with ten targets; isorhamnetin interacts with nine targets.

#### 3.2.4. Construction of PPI and Determination of Key Targets

Through the STRING database, we constructed a PPI network for DHJSD in the treatment AS. A node represents the potential target protein, and the connection between the two nodes represents the interactive relationship between the target proteins (Figure S24). The data obtained in STRING were imported into Cytoscape software to build a network (Figure S25(a)). The plug-in CytoNCA was used to calculate 47 target proteins for DC, CC, BC, EC, LAC, and NC. According to statistics, the median value of DC was 15, the median value of CC was 0.55, the median value of BC was 14.65, the median value of EC was 0.11, the median value of LAC was 8.33, and the median value of NC was 10.29. A total of 14 target proteins with all parameters greater than the median values were screened to create a subnetwork (Figure S25(b)). The plug-in CytoNCA was used again to calculate the DC, CC, BC, EC, LAC, and NC of the 14 target proteins in the subnetwork. According to statistics, the median value of DC was 23.5, the median value of CC was 0.63, the median value of BC was 61.64, the median value of EC was 0.22, the median value of LAC was 12.84, and the median value of NC was 18.13. A total of four target proteins with all parameters greater than the median values were screened to create a network (Figure S25(c)). These four target proteins are the key targets of DHJSD in the treatment of AS.

#### 3.2.5. GO Function Enrichment Analysis and KEGG Pathway Enrichment Analysis

The GO function enrichment analysis of 47 overlapping target proteins yielded 1596 entries, including 1449 BPs, 26 CCs, and 121 MFs. BP mainly involves response to lipopolysaccharide, response to molecules of bacteria, fatty acid metabolic process, and cellular response to biotic stimulus. CC mainly involves the external side of the plasma membrane, the nuclear envelope, the nuclear membrane, and the secretory granule lumen. MF mainly involves heme binding, tetrapyrrole binding, DNA-binding transcription factor binding, and nuclear receptor activity. According to *P* < 0.05, the top 10 different biological processes were selected for visual display (Figure 2). KEGG functional enrichment analysis revealed 110 pathways, of which AS-related pathways mainly involved the IL-17 signaling pathway, the TNF signaling pathway, and the rheumatoid arthritis signaling pathway. According to *P* < 0.05, the top 20 signaling pathways were selected for visual display (Figure 3).

## 4. Discussion

DHJSD is an effective prescription for treating both liver and kidney deficiency and insufficiency of qi and blood [25]. In the prescription, Radix Angelicae Pubescentis, Radix Saposhnikoviae, Radix Gentianae Macrophyllae, Cortex Cinnamomi, and Herba Asari expel wind, dampness, and cold and relieve pain [26]; Panax Ginseng, Poria Cocos, Radix Glycyrrhizae, Radix Angelicae Sinensis, Radix Rehmanniae Preparata, Radix Paeoniae Alba, and Rhizoma Chuanxiong invigorate the spleen and qi, enrich the blood, and promote blood circulation [27]; Cortex Eucommiae Ulmoidis, Radix Achyranthis Bidentatae, and Herba Taxilli detoxify the kidneys and provide nourishing essences that strengthen muscles and bones [15].

We identified the active compounds and target genes of DHJSD through TCMSP. Then, 178 candidate target genes of DHJSD that are active in AS were identified, and the key compounds of DHJSD that act on AS were screened. The main key compounds are quercetin, kaempferol, licochalcone A, and isorhamnetin. Quercetin has pharmacological effects as an antioxidant and an anti-inflammatory, it protects bones and joints, it acts as an antiapoptosis agent, it inhibits osteoclast absorption, and it regulates immune function [28–30]. Quercetin can inhibit the proliferation of the proinflammatory cytokine TNF-*α* and the gene levels of human peripheral blood mononuclear cells, it can reduce the expression of IL-1*β*, IL-6, and other inflammatory factors and matrix metalloproteinases, and it inhibits the production of inflammatory mediators, thereby improving inflammatory symptoms [28–30]. Kaempferol downregulates matrix metalloproteinases, tartrate-resistant acid phosphatase, and integrin *β*3; it inhibits the expression levels of osteoclast bone resorption-related proteins and genes and the proliferation and differentiation of monocyte macrophages into osteoclasts; and it has a bone protective effect [31, 32]. In addition, kaempferol can also reduce the activity of FGFR3, inhibit the activation level of basic fibroblast factor (bFGF) on the FGFR3-RSK2 signal axis, regulate the proliferation and migration of synovial cells and *T* cell-mediated inflammatory cytokine (IL-7, IL-21, TNF-*α*) release, and alleviate inflammation [31, 32]. Licochalcone A can delay the progression of inflammation by inhibiting the inflammatory response and inhibiting the degradation of cartilage matrix [33]. As a direct derivative of quercetin, isorhamnetin has good anti-inflammatory, antioxidant, and antiallergic effects [34, 35]. Experiments show that isorhamnetin can inhibit the NF-*k*B signaling pathway, inhibit the release of cytokines (TNF-a, IL-6, IL-1B), and alleviate inflammation [36].

PPI network analysis shows that DHJSD can affect AS through multiple targets. The main targets are CXCL8, PTGS2, VEGFA, and STAT3. The Entrez Gene summary of the CXCL8 gene shows that the protein encoded by this gene is a member of the CXC chemokine family and is the main mediator of the inflammatory response [37, 38]. A profile consisting of high levels of CXCL8 is associated with increased disease activity in AS [38]. Studies have shown that CXCL8 changes local vascular permeability in rheumatoid arthritis and that it changes the adhesion of neutrophils and endothelial cells. It causes neutrophils to accumulate at the inflammation site to cause an inflammatory reaction that ultimately results in the destruction of articular cartilage and bone [39, 40]. The expression changes of VEGF are closely related to the processes of synovial inflammation, chondrocyte apoptosis, and cartilage degeneration [41–43]. On the one hand, the proliferation and migration of VEGF lead to bone and cartilage damage [44, 45], while the increase in serum VEGF levels breaks the balance of bone metabolism in the body, inhibits bone resorption, enhances bone formation, and eventually leads to fibrosis and ossification of the sacroiliac joints, spine and nearby tendons, the ligament-bone attachment points, and new bone formation [46]. PTGS2 is also known as cyclooxygenase 2, and this gene serves as an important target in the inflammation process, which can convert arachidonic acid into PGH2 and cause inflammation [47]. STAT3 regulates the polarization state of macrophages, promotes their transformation into M2 type, promotes the secretion of anti-inflammatory cytokines and cell growth factors, has anti-inflammatory effects, and promotes bone repair functions [48]. In addition, activation of the STAT3 signaling pathway can promote the proliferation of bone morphogenetic protein 2, which binds to its corresponding receptor to mediate the osteogenic differentiation of bone marrow mesenchymal cells and the calcification of osteoblasts [49].

During the GO enrichment analysis in this study, it was discovered that the biological process of DHJSD in the treatment of AS includes responses to lipopolysaccharides, to molecules of bacterial origin, to fatty acid metabolic processes, to the external side of plasma membranes, to the nuclear envelope, to the nuclear membrane, to heme binding, to tetrapyrrole binding, to DNA-binding, to transcription factor binding, and to many other biological processes. These biological processes play a key role in the treatment of AS by DHJSD.

KEGG enrichment pathway analysis showed that many pathways were closely related to the pathogenesis of AS. The main pathways included the IL-17 signaling pathway, the TNF signaling pathway, and the rheumatoid arthritis signaling pathway. The IL−17 signaling pathway and the TNF signaling pathway play a central role in the pathogenesis of AS [50]. Mouse models show that changes in these pathways affect the development and severity of inflammation [51, 52]. These results indicate that DHJSD acts on AS in a variety of ways. The key pathways and target genes in the pathway are worthy of further study.

Meta-analysis is a systematic, quantitative, and comprehensive statistical method based on previous research results. It is often used to evaluate interventional RCTs in evidence-based medicine to objectively evaluate clinical efficacy. Therefore, in this study, we compiled current evidence on the overall effect of DHJSD on AS in 860 patients from 10 studies. The results of the meta-analysis showed that DHJSD treatment of AS has clinical efficacy with a reduced occurrence of adverse reactions. Evidence-based medicine methods show the efficacy of DHJSD treatment on AS at the clinical level, which is more meaningful than experimental verification. Through the integration of meta-analysis and network pharmacology analysis, we successfully determined the clinical efficacy of DHJSD in the treatment of AS and the targets, components, and pathways of DHJSD in the treatment of AS.

However, this study also includes some other limitations. First, due to the particularity of traditional Chinese medicine decoctions, it is difficult to implement allocation concealment and blinding. Second, pharmacological analysis is mainly used to demonstrate the synergistic effects of herbal chemical components obtained through existing databases, rather than experimental verification, which needs to be further verified in future studies.

## 5. Conclusions

According to existing research data, DHJSD treatment of AS can improve clinical efficacy and reduce adverse reactions. Its mechanism of action works mainly through its active ingredients, such as quercetin, kaempferol, licochalcone A, and isorhamnetin, which act on key target genes such as CXCL8, PTGS2, VEGFA, and STAT3, thereby regulating the IL-17 signaling pathway, the TNF signaling pathway, the rheumatoid arthritis signaling pathway, and other related signaling pathways. DHJSD should eventually be given a formal role in the treatment of AS.

## Figures and Tables

**Figure 1:** Risk of bias summary.

**Figure 2:** Ten most significant therapy target genes of DHJSD on AS based on Gene Ontology analysis.

**Figure 3:** Twenty most significant therapy target genes of DHJSD on AS based on pathway enrichment analysis.

**Table 1:** Demographic and clinical characteristics of the included studies.

Author, year	Sample size (I/C)	Age (years) (I/C)	Intervention	Control	Period of treatment
Sun et al., [15]	55/56	33.6 ± 12.9/34.4 ± 13.2	Duhuo Jisheng Decoction	Meloxicam tablets + sulfasalazine tablets	4 m
Zhang et al., [16]	58/60	18–45/13–48	Duhuo Jisheng Decoction	Naphtobumethone tablets + sulfasalazine tablets	1 m
Dong [17]	50/50	35.62 ± 9.53/36.32 ± 9.66	Duhuo Jisheng Decoction	Meloxicam tablets + sulfasalazine tablets	1 m
Yan et al., [18]	32/28	37.54 ± 13.67/38.25 ± 12.94	Duhuo Jisheng Decoction	Indometacin + sulfasalazine tablets	2 m
Pan et al., [19]	39/39	33 ± 15/36 ± 14	Duhuo Jisheng decoction	Meloxicam tablets + sulfasalazine tablets	2 m
Yu et al., [20]	52/40	33.28 ± 5.27/32.16 ± 4.89	Duhuo Jisheng decoction	Diclofenac sodium + sulfasalazine tablets	24 w
Zuo et al., [21]	42/45	33.76 ± 6.74/32.83 ± 7.12	Duhuo Jisheng decoction	Methotrexate tablets + sulfasalazine tablets	3 w
Lu [22]	30/30	43.23 ± 4.10/42.12 ± 4.01	Duhuo Jisheng decoction	Meloxicam tablets + sulfasalazine tablets	3 m
Zhou [23]	36/31	18–50/17–49	Duhuo Jisheng decoction	Indometacin + sulfasalazine tablets	3 m
Yang [24]	42/45	33.76 ± 6.74/32.83 ± 7.12	Duhuo Jisheng decoction	Methotrexate tablets + sulfasalazine tablets	3 m

I, intervention; C, control; M, month; W, week.

**Table 2:** Results of meta-analysis of each outcome indicator.

Outcome indicator	The number of studies	The number of patients	Association test			Heterogeneity		
			RR/SMD	95% CI	*P* val	Model	*P* val	I2
The clinical effective rate	10	858	**RR = 1.30**	**(1.16, 1.44)**	**<0.00001**	Random	0.02	53%
BASFI	4	385	SMD = −0.46	(−1.77, 0.85)	0.49	Random	<0.00001	97%
BASDAI	3	285	SMD = −0.36	(−1.95, 1.23)	0.66	Random	<0.00001	97%
VAS score	6	515	**SMD = −0.79**	**(−1.19, −0.40)**	**<0.0001**	Random	0.0003	97%
Finger-to-floor distance	5	481	**SMD = −1.55**	**(−2.66, −0.44)**	**0.006**	Random	0.00001	97%
Morning stiffness time	3	230	**SMD = −1.23**	**(−2.21, −0.25)**	**0.01**	Random	<0.0001	91%
Degree of motion of chest	3	285	**SMD = 0.24**	**(0.01, 0.47)**	**0.04**	Fixed	0.80	0%
Schober's test values	3	321	**SMD = 0.23**	**(0.01, 0.45)**	**0.04**	Fixed	0.24	31%
ESR	9	800	**SMD = −1.07**	**(−1.69, −0.46)**	**0.0006**	Random	<0.00001	94%
CPR	7	582	**SMD = −2.31**	**(−3.52, −1.10)**	**0.0002**	Random	<0.00001	97%
BALP	2	211	SMD = 0.18	(−0.36, −0.71)	0.51	Random	0.05	74%
IL-6	2	211	**SMD = −1.72**	**(−3.06, −0.38)**	**0.01**	Random	<0.0001	94%
BGP	2	211	SMD = 3.14	(−1.62, 7.89)	0.20	Random	<0.00001	99%
Incidence of gastrointestinal events	5	446	**RR = 0.27**	**(0.13, 0.54)**	**0.0002**	Fixed	0.62	0%
Incidence of skin events	5	446	**RR = 0.13**	**(0.03, 0.48)**	**0.002**	Fixed	0.88	0%
Incidence of abnormal liver function	6	522	**RR = 0.28**	**(0.11, 0.67)**	**0.004**	Fixed	0.85	0%
Incidence of abnormal renal function	3	292	RR = 0.29	(0.05, 1.72)	0.17	Fixed	0.96	0%

RRs, risk ratios; CIs, confidence intervals; SMD, standard mean difference; ESR, erythrocyte sedimentation rate; CPR, C-reactive protein; IL-6, interleukin 6; VAS, visual analog scale; BASFI, Bath Ankylosing Spondylitis Functional Index; BASDAI, Bath Ankylosing Spondylitis Disease Activity Index; BGP, bone Gla-containing protein; BALP, bone alkaline phosphatase.

## Data Availability

The data used to support the findings of this study are available from the corresponding author upon request.

## Abbreviations

TCMSP: Traditional Chinese Medicine Systems Pharmacology
NCBI: National Center For Biotechnology Information
OMIM: Online Mendelian Inheritance In Man
PharmGKB: Pharmacogenomics Knowledgebase
TTD: Therapeutic target database
DHJSD: Duhuo Jisheng Decoction
AS: Ankylosing spondylitis
GO: Gene ontology
KEGG: Kyoto Encyclopedia of Genes and Genomes
PPI: Protein-protein interaction
ESR: Erythrocyte sedimentation rate
CPR: C-reactive protein
IL-6: Interleukin 6
VAS: Visual analog scale
BASFI: Bath Ankylosing Spondylitis Functional Index
BASDAI: Bath Ankylosing Spondylitis Disease Activity Index
BGP: Bone Gla-containing protein
BALP: Bone alkaline phosphatase
RRs: Risk ratios
CIs: Confidence intervals
SMD: Standard mean difference
BC: Betweenness centrality
CC: Closeness centrality
DC: Degree centrality
EC: Eigenvector centrality
LAC: Local average connectivity-based method centrality
NC: Network centrality
BP: Biological process
CC: Cellular component
MF: Molecular function.

## Supplementary Materials

Supplementary Materials Figure S1: flowchart of selection process. Figure S2: forest plot of DHJSD treatment versus control for clinical effective rate. Figure S3: forest plot of DHJSD treatment versus control for BASFI. Figure S4: forest plot of DHJSD treatment versus control for BASDAI. Figure S5: forest plot of DHJSD treatment versus control for VAS score. Figure S6: forest plot of DHJSD treatment versus control for finger-to-floor distance. Figure S7: forest plot of DHJSD treatment versus control for morning stiffness time. Figure S8: forest plot of DHJSD treatment versus control for degree of motion of chest. Figure S9: forest plot of DHJSD treatment versus control for Schober's test. Figure S10: forest plot of DHJSD treatment versus control for ESR level. Figure S11: forest plot of DHJSD treatment versus control for CPR level. Figure S12: forest plot of DHJSD treatment versus control for BALP level. Figure S13: forest plot of DHJSD treatment versus control for IL-6 level. Figure S14: forest plot of DHJSD treatment versus control for BGP level. Figure S15: forest plot of DHJSD treatment versus control for incidence of gastrointestinal events. Figure S16: forest plot of DHJSD treatment versus control for incidence of skin events. Figure S17: forest plot of DHJSD treatment versus control for incidence of abnormal liver function. Figure S18: forest plot of DHJSD treatment versus control for incidence of abnormal renal function. Figure S19: forest plot of subgroup analysis on clinical effective rate. Figure S20: sensitivity analysis of all the studies assessing clinical effective rate. Figure S21: Begg's funnel plot of clinical effective rate. Figure S22: Venn diagram of DHJSD-related targets and AS-related targets. Figure S23: “DHJSD-active compounds-target genes-AS” network. Figure S24: PPI network of DHJSD acting on AS. Figure S25: hub genes acquired from the PPI network (BC = betweenness centrality, CC = closeness centrality, DC = degree centrality, EC = eigenvector centrality, LAC = local average connectivity-based method centrality, and NC = network centrality). Table S1: information of active compounds and corresponding target number of Duhuo Jisheng Decoction.
